# Improving Recognition of Overlapping Activities with Less Interclass Variations in Smart Homes through Clustering-Based Classification

**DOI:** 10.1155/2022/8303856

**Published:** 2022-06-02

**Authors:** Muhammad Usman Sarwar, Labiba Fahad Gillani, Ahmad Almadhor, Manoj Shakya, Usman Tariq

**Affiliations:** ^1^Department of Computer Science, National University of Computer and Emerging Sciences, Islamabad, Pakistan; ^2^College of Computer and Information Sciences, Al Jouf University, Sakakah, Saudi Arabia; ^3^Department of Computer Science and Engineering, Kathmandu University, Dhulikhel, Nepal; ^4^College of Computer Engineering and Sciences, Prince Sattam Bin Abdulaziz University, Al-Kharj, Saudi Arabia

## Abstract

The systems of sensing technology along with machine learning techniques provide a robust solution in a smart home due to which health monitoring, elderly care, and independent living take advantage. This study addresses the overlapping problem in activities performed by the smart home resident and improves the recognition performance of overlapping activities. The overlapping problem occurs due to less interclass variations (i.e., similar sensors used in more than one activity and the same location of performed activities). The proposed approach overlapping activity recognition using cluster-based classification (OAR-CbC) that makes a generic model for this problem is to use a soft partitioning technique to separate the homogeneous activities from nonhomogeneous activities on a coarse-grained level. Then, the activities within each cluster are balanced and the classifier is trained to correctly recognize the activities within each cluster independently on a fine-grained level. We examine four partitioning and classification techniques with the same hierarchy for a fair comparison. The OAR-CbC evaluates on smart home datasets Aruba and Milan using threefold and leave-one-day-out cross-validation. We used evaluation metrics: precision, recall, *F* score, accuracy, and confusion matrices to ensure the model's reliability. The OAR-CbC shows promising results on both datasets, notably boosting the recognition rate of all overlapping activities more than the state-of-the-art studies.

## 1. Introduction

Independent living has attracted increasing attention to ubiquitous computing (e.g., developing inexpensive wireless sensors besides efficient data processing techniques) [1–6]. These techniques help in the development of low-cost and technology-driven healthcare solutions for elderly people [7–13]. According to a survey in Norway in 2016, people aged between 67 and 79 years are 10.4% of the population, and the age of more than 80 years is 4.2% [14]. Furthermore, by 2060, this age group of 60–80 will become almost 19%. The increase in the old age population also concerns other European countries and China, the United States, Korea, and Japan.

A smart home (SH) is a housing situation enriched with the diversity of multi-model sensors, devices, actuators, and information and communication technology (ICT)-based services and systems. To support independent living in SH, the environmental changes are monitored, and residents' activities are detected. An assisted living system can process through observed sensor data to make timely decisions and take appropriate actions to support independent living [15].

The most widely used SH projects with physical test beds for activity recognition are the MavHome project [16], CASAS project [17], Georgia Tech aware home [18], and Gator Tech Smart House [19]. Researchers are now concerned about applying smart environment technology in healthcare assistance based on these advancements.

In smart homes, the activities, i.e., toileting, meal preparation, and dish washing, are performed, and their readings are collected from switch sensors embedded on different objects (i.e., cupboard, fridge, oven, and stove). The participants have different lifestyles and abilities to perform activities of daily living (ADLs) in SH. Although the ADLs follow some sort of sequence types, there are no strict rules on the sequence (e.g., in tea preparation, first the stove is turned on and then the kettle is placed or vice versa) and duration of the specific actions to perform activities [16, 20]. Thus, the diverse range of ADLs, variations, and performing styles required a generalized approach and handled these variations in recognition.

Modern research for activity recognition focused on the use of probabilistic and statistical analysis methods to train the activity models [7, 21–26]. Moreover, some researchers also focused on techniques that are generally logical or ontological and used domain knowledge with priory heuristics as a base to create activity models [15, 27–30]. Researchers also considered clustering techniques where the activity data are not labeled properly.

### 1.1. Problem Statement

Activity recognition is a challenging problem as the assisted living is now shifted towards cognitive ADL assistance [28, 31–33]. Cognitive ADL assistance means providing on-time guidance and support to elderly people and people with cognitive impairments. Since every use has their preferences in performing an activity, thus resulting in dintinct activity instances (e.g., in tea prepration, a user may first turn on the stove and then place the kettle on stove or vice versa) [16, 20]. However, activities performed in the exact location share similar features and have fewer interclass variations due to which overlapping problem occurs, thus affecting the reliability of the healthcare system. The most overlapping activities are dish wash, meal preparation, enter home, and leave home in the Aruba [7] dataset and bed to toilet, morning medicine, and evening medicine in the Milan [34] dataset. The diversity of ADLs, minor variations, and performing styles require an approach generalized to large-scale activity modeling and recognition.

Our focus is on exploring overlapping activities with fewer interclass variations and improving their recognition performance in this research work. For this objective, we propose a generic overlapping activity recognition model using clustering-based classification (OAR-CbC). The highlighted contributions of this study are summarized as follows: we proposed a two-layer generic clustering-based classification activity recognition model. We analyzed that soft clustering methods (fuzzy C-means [35]) makes better clusters than the complex clustering methods (*K*-means [36] and DBSCAN [37]) for this particular problem while balancing the clusters adds further improvements. We improved the performance in terms of precision, recall, and F score of all overlapping activities that share similar features among the existing systems that used the same dataset.

The rest of the study is organized as follows: Section 2 discusses the related work on activity recognition and its techniques.  Section 3 demonstrates the proposed methodology.  Section 4 provides the experimental setup, evaluation measures, detailed results, and comparison with state-of-the-art research. Finally, Section 5 summarizes this article and provides the future directions.

## 2. Literature Review

Many assisted living approaches are proposed based on smart homes and collected datasets with the advancement in ubiquitous computing. The smart home dataset collects sensor events and trains the activity model to map the relationship between the events and the activities. The activity model is then used to predict the future recognition of the events. The learning method SVM is applied to find differences between the correct and incorrect assignments [21]. They find the underlying distribution through clustering within each activity class, and the confidence score is measured to reduce the false-positive rate of the assigned category. The resampling method bootstrap is also used to improve the data representation in the training where the number of instances is limited in a cluster. The performance metrics show that their results are comparatively better than other approaches, but the accuracy is less for overlapping datasets because of significantly fewer interclass variations.

The proposed approach [22] is based on Dempster–Shafer's theory. The fusion of contextual information that is collected from sensor data is used. The approach can distinguish different activities. Comparing the results of naive Bayes, HMM, and conditional random fields makes a hypothesis that a generalized model can be developed for everyday activities that can model multiple environment settings and resident types by the semi-supervised approach [7]. A general model is trained with less semi-supervised data by combining latent Dirichlet allocation (LDA) and AdaBoost. For misclassification, a combination of AdaBoost, HMM, and CRF is used to explore the temporal information in the data. The proposed approach is inspired by the claim that performing activities is dependent on age, gender, and other physical characteristics of different people [38]. The study [23] proposed an approach to recognize highly overlapping human daily life activities. They introduced a two-layer framework for coarse-grained and fine-grained level recognition. The coarse-grained recognition identifies whether the activity is high-overlapping or not. An output of the coarse-grained classification becomes the input to the fine-grained classification, which classifies the activity labels.

An unobtrusive approach is proposed using the deep convolutional network and binary sensors for activity recognition [39]. The binary state sensor reading is converted into images using different sliding window techniques. For activity classification, a deep convolutional neural network was applied. The study [40] proposed a clustering-based classification approach that is efficient for boosting the accuracy by recognizing similar activities on a fine-grained level. They identify the significant features and reduce the feature dimensions using principle component analysis (PCA) feature selection method. Then, they group similar activities using Lloyd's clustering algorithm. To recognize the labels of the activities, the combination of *K*-nearest neighbors (KNNs) with Dumpster–Shafer theory (DST) of evidence, the evidence theoretic *K*-nearest neighbors (ET-KNNs), is used. Authors in [15] proposed an unsupervised learning technique for discovering and activities from sensor data collected from CASAS smart home project.

The hidden Markov model (HMM) represents the activities and recognizes those activities when performed. A similar approach for activity recognition based on ontological modeling and semantic reasoning is proposed by [20]. They analyzed the nature and characteristics of ADLs. The proposed algorithm can support coarse-grained and fine-grained level activity recognition. The proposed approach overcomes the flexibility issues that conventional logical approaches have faced using inflexible activity representations. An active learning approach is proposed based on the hypothesis that sensors frequently fired together simultaneously with similar duration represent a daily activity. If these groups detect automatically from the raw sensor firings, then users have just labeled each group as an activity, and all the instances of this group can be automatically labeled [27].

An intention recognition technique is proposed, in which environmental sensors are used to identify the intention of the inhabitant based on the object usage [28]. Using an ontology, a library of goal hierarchy is encoded where sensor activation performed by inhabitant represented atomic actions. They consider the current atomic and related actions within a specific interval for a predictive reasoning technique to determine the most expected goal of the inhabitants. In the study, [41], four significant tasks, data acquisition, feature extraction, activity discovery, and activity recognition, were performed. The wireless body sensor networks (WBSNs) are used for body monitoring. The cloud-assisted agent-based smart home environment (CASE) includes three-layered architecture responsible for sensing and actuating. Managers of this framework are agents that manage actuators, sensors, and complex algorithms locally and on the cloud. Both the fixed sensors data and mobile sensors data are used to identify the complex activities of inhabitants.  Table 1 shows the summary of the existing research approaches.

To the best of our knowledge, researchers [21, 23, 39, 40] used the machine learning approaches such as NBC [7], HMM [38], ontological [28], and Dempster–Shafer theory [22] for activity recognition but do not consider overlapping activities primarily. The probabilistic approach with ensemble methods [38] is also not efficient because it boosts only the overall accuracy while unable to improve the recognition rate of overlapping activities. Thus, reliability is a significant concern when recognition has to apply to real-time systems, i.e., health monitoring.

## 3. Proposed OAR-CbC Approach

In this research work, we focus on exploring the recognition of overlapping activities or activities with less interclass variations on coarse-grained and fine-grained levels by a two-layer clustering-based classification model. To deal with the overlapping problem, we apply the clustering method to accurately group activities on a coarse-grained level, balance the activities within each cluster, and then use the classification method to recognize the activities on a fine-grained level. Some activities have fewer interclass variations, e.g., dish wash, meal preparation, enter home, and leave home in the Aruba [7] dataset and bed to toilet, morning medicine, and evening medicine in the Milan [34] dataset. Our proposed approach OAR-CbC consists of four steps: feature extraction, clustering, data balancing, and classification. The model's performance is assured by different metrics: accuracy, precision, F score, and recall. Our approach is novel and better than the state-of-the-art work.  Figure 1 demonstrates our proposed approach.

### 3.1. Feature Extraction

First, the features are extracted from the pre-segmented dataset: Milan [34] and Aruba [7]. Because these datasets contain raw sensor readings, as shown in Figure 2, the feature matrix is extracted to input the model. First, 33 unique features (based on the sensor used) and one label, the name of activities, are extracted from the Milan dataset for all 15 types of activities. Then, the duration feature, the total time to complete an activity, is extracted by subtracting the time of the first sensor reading when the activity started from the last reading and when the activity ends. The duration feature values are then converted into seconds. For each activity instance, the frequency of each sensor is summed. The feature matrix of the Milan dataset contains 34 features with the activity label. Similarly, 40 unique features are used in all 11 types of activities for the Aruba dataset, and a duration feature is extracted. The sensor readings, which were not annotated within the start and end of an activity, are ignored.

### 3.2. Clustering

We are dealing with a similar set of feature problem, and there is significantly less discriminating information between activities; therefore, it is important to address the interclass activity variations. The activities are grouped to get the maximum variance for interclass activities. Applying this two-layered model (i.e., clustering and classification) is to recognize the confusing activities (i.e., overlapping activities) on the fine-grained level. The single-layer model (i.e., classification) cannot adaptively recognize overlapping activities. Moreover, it adopts multichannel processing. The more accurate the grouping (clustering) is, the more accurately it recognizes similar activities. After extraction of features, the fuzzy C-means [35] clustering technique is applied to group similar activities into clusters. The detail of fuzzy C-means and its parameter is explained below. Also, for analysis and comparison purposes, other three clustering techniques are applied namely hierarchical [42], *K*-mean [36], and DBSCAN [37]. These four techniques are applied because the cluster's shape depends on data, and it is important to know the exact grouping of data. Fuzzy C-means is the soft clustering technique and would make better clusters than the hierarchical *K*-means and DBSCAN, as these are the hard clustering techniques.

### 3.3. Fuzzy *C*-Means

The authors in [35] initially proposed the fuzzy C-means clustering (FCM) algorithm. It was improved by Bezdek [43] in 1981. The fuzzy C-means algorithm works by calculating the similarity based on the membership values of each activity instance with respect to each activity type. It is one of the most popular and widely used fuzzy clustering algorithms. Below, the working of the fuzzy C-means algorithm is explained.

- Initialize number of clusters *C*(2 ≤ *C* < *n*)
- Set a value for fuzziness parameter (*m*)
- Assign coefficients randomly to each data point for being in the clusters
- Calculate the centroid each cluster as shown in (1)
- Compute again its coefficients of being in the clusters for each node

(1) $$\begin{array}{c} c_{k}=\frac{\sum_{x}w_{k}{\left(x\right)}^{m}x}{\sum_{x}w_{k}{\left(x\right)}^{m}}, \end{array}$$

where *m* is the hyper-parameter that controls the fuzziness. Given an input matrix *X*=*x*_1_, *x*_2_,…, *x*_*n*_, the fuzzy *C*-mean algorithm works to minimize an objective function. Below describes the object function:

(2) $$\begin{array}{c} \underset{C}{\arg\min}\sum_{i=1}^{n}\sum_{j=1}^{c}w_{ij}^{m}{\left\|x_{i}-c_{j}\right\|}^{2}, \end{array}$$

where

(3) $$\begin{array}{c} w_{ij}=\frac{1}{\sum_{k=1}^{c}{\left(\left\|x_{i}-c_{j}\right\|/\left\|x_{i}-c_{k}\right\|\right)}^{2/m-1}}, \end{array}$$

where *w*_*ij*_ represents the degree to which element *x*_*i*_ belongs to cluster *c*_*j*_.

## 4. Data Balancing

The data imbalance in similar activities could create ambiguity, and the activity with the majority occurrence would take advantage. At the same time, the recognition rate of activity with fewer instances is decreased [44]; e.g., the “Meal Preparation” activity performed more than “Dish Washes” in the Aruba dataset [7]. Also, after clustering, the activity with fewer instances may be distributed in more than one cluster (i.e., “House Keeping” has only 33 instances and could be distributed as 20 and 13 in two clusters). Therefore, an over-sampling technique, synthetic minority over-sampling technique (SMOTE) [44], is applied to each cluster of all the four clustering techniques independently to balance the instances of the activities. It takes the input of which activity Ai to balance and at what rate *N*% it has to balance and *K* as nearest neighbor. For every instance, SMOTE first calculates the distance between the original instance and the selected *K*-nearest neighbors and then multiplies the distance with the range between 0 and 1. The nearest neighbors are to be chosen, and we use the three nearest neighbors for the “Resperate” activity in the Aruba dataset because it has only six instances. For example, if we want to over-sample 200% the “Resperate” activity, then three nearest neighbors from 6 instances are chosen randomly, and doubles of the six instances are created.

### 4.1. Classification

After grouping similar activities using fuzzy C-means and data balancing, we implement artificial neural network (ANN) [45] with different parameter settings. The classifier applies to each cluster independently and then calculates the average of each evaluation metric of all the clusters concerning the activities; e.g., if the “Work” activity comes in 3 clusters, then the average precision of these 3 clusters is calculated according to “Work” activity. The parameters are also tuned to conclude the best performance of one of them. Also, some other classifiers are implemented, and the performance of each is compared. These included sequential minimal optimization (SMO) [46], evidence theoretic *K*-nearest neighbor (ET-KNN) [47], and *K*-nearest neighbor (KNN) [48]. Each classifier gives a different result according to clustering techniques. The ANN is more robust than all other classifiers to the best of our knowledge, as shown in the result section. Below is the detail of the classifier.

### 4.2. Artificial Neural Network (ANN)

An ANN consists of at least three layers of nodes: an input layer, a hidden layer, and an output layer [45]. Each node is taken as a neuron, which uses a nonlinear activation function as explained in (4). It uses backpropagation for training. Below is the equation that illustrates the working:

(4) $$\begin{array}{c} y\left(v_{i}\right)=\tan h\left(v_{i}\right), \end{array}$$

(5) $$\begin{array}{c} Ε\left(n\right)=\frac{1}{2}\sum_{j}e_{j}^{2}\left(n\right). \end{array}$$

The node weights are adjusted based on corrections as explained in (5) that minimize the error in the entire output.

## 5. Experimental Setup

This section explains the used dataset, how the experiments are carried out, and different evaluation measures that ensure the proposed approach's reliability.

### 5.1. Dataset

The dataset of Milan [34] contains sensor data that were collected in the home of a volunteer adult. The residents in the home were a woman and a dog. The woman's children visited on several occasions. The 15 activities annotated within the dataset are shown in Table 2. The activities “Bed to Toilet” with “Master Bathroom” and “Morning Medicine” with “Evening Medicine” are the most overlapping in this dataset. Similarly, the Aruba [7] dataset contains 11 activities also shown in Table 2. The “Wash Dishes” with “Meal Preparation” and “Enter Home” with “Leave Home” are the most overlapping activities in this dataset. Table 2 shows the summary of both dataset. Figure 2 shows the notations used for each feature such as sensor IDs where motion sensor is represented by “M,” door sensor is represented by “D,” and temperature sensor is represented by “T.” It also shows two states of sensors: On or off. This sample annotation shows that the participant was watching Tv.

### 5.2. Evaluation Performance Metrics

The proposed approach is evaluated on Milan and Aruba datasets using threefold cross-validation and leave-one-day-out cross-validation. The threefold cross-validation works by leaving 1 : 3 part of the data for testing and using 2 : 3 part of the data for training. In leave-one-day-out cross-validation activities are performed as one day used for testing and remaining for training until all data are used for testing once day by day as the Aruba dataset contains data of 220 days, so a total of 220-folds would be built for each classifier. Precision, recall, *F* score, and accuracy are used as performance metrics for comparison. For each activity class Ai, true positive (TP) is the number of examples correctly recognized as Ai and false negative (FN) is instances of activity Ai that incorrectly recognized as other activity classes Aj. Further, true negative (TN) is the instances correctly recognized as not from that activity Ai. False positive (FP) is the activity instances that belong to other activity classes but are recognized as Ai. Recall that is also called sensitivity or true-positive rate is the ratio of correctly labeled activity instances Ii,…, In out of total instances In of that activity Ai. Precision is the rate of correctly labeled instances Ii,…, In from the total instances of a class Ai, whereas *F*1 score is the weighted average of precision and recall in the range of 0-1, where 0 shows the worst performance and 1 shows the best performance.

Recall is given as follows:
  (6) $$\begin{array}{c} \text{Recall}=\frac{\text{TP}}{\text{TP}+\text{FN}}. \end{array}$$
Precision is given as follows:
  (7) $$\begin{array}{c} \text{Precision}=\frac{\text{TP}}{\text{TP}+\text{FP}}. \end{array}$$
Accuracy is given as follows:
  (8) $$\begin{array}{c} \text{Accuracy}=\frac{\text{TP}+\text{TN}}{\text{TP}+\text{TN}+\text{FP}+\text{FN}}. \end{array}$$
*F* measure is given as follows:
  (9) $$\begin{array}{c} F-\text{Measure}=2\times \frac{\text{Precision}\times \text{Recall}}{\text{Precision}+\text{Recall}}. \end{array}$$

## 6. Result Analysis

The primary focus of this research is on clustering methods because the best choice of clustering technique that makes more reliable clusters of similar activities can improve the performance of recognition. Also, activities balancing the activities can handle less discriminated information between overlapping activities, i.e., “Meal Preparation” and “Wash Dishes” in Aruba dataset. Below, the fuzzy C-means, hierarchical, *K*-means, and DBSCAN clustering techniques concerning the ANN, ET-KNN, KNN, and SMO classifiers are shown. In addition, an analysis before and after balancing the activities within each cluster is also performed. To the best of our knowledge, a combination of fuzzy C-means and ANN gives a higher recognition rate of almost 85% without activities balancing and 94% with activities balancing on the Aruba dataset.

### 6.1. Results without Activities Balancing

The results without activities balancing all the four classifiers concerning the four clustering techniques using threefold and leave-one-day-out cross-validation on the Aruba and Milan datasets are shown in this section. The complete analysis is shown in Table 3 for the Aruba dataset.

Table 3 shows the results on the Aruba dataset using threefold cross-validation. It demonstrates that the combination of fuzzy C-means with ANN achieved 2%, 2%, and 4% higher *F* score than the hierarchical, *K*-means, and DBSCAN in combination with ANN. The ET-KNN and KNN classifier in combination with fuzzy C-means achieved 1%, 2%, and 3% better *F* score than the combination of ET-KNN and KNN with hierarchical, *K*-means, and DBSCAN, while the SMO in combination with hierarchical achieved 1%, 2%, and 2% higher *F* score than the SMO in combination with fuzzy C-means, *K*-means, and DBSCAN, respectively.

Table 4 shows the results on the Milan dataset using threefold cross-validation. The combination of fuzzy C-means with ANN achieved 2%, 4%, and 4% higher *F* score than the combination of hierarchical, *K*-means, and DBSCAN with ANN. ET-KNN with fuzzy C-means achieved 2%, 3%, and 4% higher *F* score than the combination of ET-KNN with hierarchical, *K*-means, and DBSCAN. The combination of KNN with fuzzy C-means also achieved 3%, 3%, and 5% higher *F* score than the combination of KNN with the hierarchical, *K*-means, and DBSCAN. Finally, the SMO combined with fuzzy C-means achieved 3%, 3%, and 3% higher *F* score than the combination of SMO with the hierarchical, *K*-means, and DBSCAN, respectively.

### 6.2. Confusion Matrix without Activities Balancing

However, the overall performance of ANN is much better than ET-KNN, KNN, and SMO when grouping similar activities with fuzzy C-means, hierarchical, *K*-means, and DBSCAN. However, the focus was on overlapping activities and required to improve the performance of that activities. The “Dish Wash” with “Meal Preparation,” “Leave Home” with “Enter Home,” and “Resperate” with “Work” are the most overlapping activities in the Aruba dataset, while the “Morning Medicine” with the “Kitchen” and “Evening Medicine,” “Bed to Toilet” with “Master Bathroom,” and “Medicine” with “Morning Medicine” and “Evening Medicine” are the most overlapping activities. However, by calculating the confusion matrices, it is analyzed that overlapping activities' performance is not so much better to be considered. Below, confusion matrices 5, 6, 7, and 8 show with the bold cells how instances of overlapping activities get mixed.

Table 5 presents a confusion matrix on the Aruba dataset using threefold cross-validation in the combination of fuzzy C-means with ANN while activities are imbalanced. It shows that the activity “House Keeping” is confused with “Eating” of 10%. Almost 44% of “Wash Dish” activity instances are identified as “Meal Preparation” activity. 45% of activity “Leave Home” instances are identified as “Enter Home,” and 10% of the instances of activity “Enter Home” are identified as activity “Leave Home,” because the same door sensor is used in both activities. Also, 18% of activity “Resperate” instances are identified as activity “Work.”

Table 6 shows the confusion matrix on the Aruba dataset using threefold cross-validation in the combination of hierarchical with ANN while activities are imbalanced. The correct assignment of the “Wash Dish” activity is 45%, while 45% and 10% of instances are identified as “Meal Preparation” and “Eating” activities. 25% of activity “Leave Home” instances are identified as “Enter Home,” and 10% of “Enter Home” instances are identified as “Leave Home” because the same door sensor is used in both activities. Also, 15% of activity “Resperate” instances are identified as activity “Work.”

Table 7 shows the confusion matrix on the Milan dataset using threefold cross-validation in the combination of fuzzy C-means with ANN while activities are imbalanced. It shows that 15% of “Bed to Toilet” activity instances are recognized as “Master Bathroom.” 10% and 7% of “Morning Medicine” instances are identified as “Kitchen” and “Evening Medicine” activities because medicine would be placed in the kitchen. 15% of “Chore” instances are recognized as “Master Room” activity. 21% and 8% of “Evening Medicine” instances are identified as “Morning Medicine” and “Kitchen.” Also, 10% and 8% of “Medicine” instances are identified as “Evening Medicine” and “Morning Medicine,” respectively.

Table 8 shows the confusion matrix on the Milan dataset using threefold cross-validation in the combination of hierarchical with ANN while activities are imbalanced. It shows that 17% of “Bed to Toilet” instances are recognized as “Master Bathroom,” while 13% vice versa. 13% of “Dinner” instances are recognized as “Kitchen,” which was not confused when fuzzy C-means is used. 10% and 12% of “Morning Medicine” instances are identified as “Kitchen” and “Evening Medicine” activities. 15% of “Chore” instances are recognized as “Master Room” activity. 22% and 8% of “Evening Medicine” instances are identified as “Morning Medicine” and “Kitchen.” Also, 11% and 7% of “Medicine” instances are identified as “Evening Medicine” and “Morning Medicine,” respectively.

## 7. Results with Activities Balancing

The above tables of confusion matrices 5, 6, 7, and 8 shows with the bold cells that how instances of overlapping activities get mixed with each other. So, after applied over-sampling method SMOTE on each cluster independently with respect to all clustering techniques on both dataset, we again extract results with all four classifiers. After that, it is analyzed that with balanced activities, almost 10% higher score was achieved than imbalanced activities as shown in Tables 9–12.

Table 9 shows the results on the Aruba dataset using threefold cross-validation. It demonstrates that the combination of fuzzy C-means with ANN achieved 5%, 7%, and 10% higher *F* score than the combination of hierarchical, *K*-means, and DBSCAN with ANN. ET-KNN with fuzzy C-means achieved 2%, 4%, and 7% higher *F* score than the combination of ET-KNN with hierarchical, *K*-means, and DBSCAN. The combination of KNN with fuzzy C-means also achieved 2%, 5%, and 8% higher *F* score than the combination of KNN with the hierarchical, *K*-means, and DBSCAN, while the SMO in combination with fuzzy C-means achieved 1%, 5%, and 4% higher *F* score than the combination of SMO with the hierarchical, *K*-means, and DBSCAN, respectively.

Table 10 shows the results on the Aruba dataset using leave-one-day-out cross-validation. It demonstrates that the combination of fuzzy C-means with ANN achieved 5%, 7%, and 9% higher *F* score than the combination of hierarchical, *K*-means, and DBSCAN with ANN. ET-KNN with fuzzy C-means achieved 1%, 3%, and 7% higher *F* score than the combination of ET-KNN with hierarchical, *K*-means, and DBSCAN. The combination of KNN with fuzzy C-means also achieved 1%, 5%, and 7% higher *F* score than the combination of KNN with the hierarchical, *K*-means, and DBSCAN, while the SMO in combination with fuzzy C-means and hierarchical achieved 4% and 3% higher *F* score than the combination of SMO with the *K*-means and DBSCAN, respectively.

Table 11 shows the results on the Milan dataset using threefold cross-validation. It demonstrates that the combination of fuzzy C-means with ANN achieved 3%, 7%, and 9% higher *F* score than the combination of hierarchical, *K*-means, and DBSCAN with ANN. ET-KNN with fuzzy C-means achieved 1%, 3%, and 6% higher *F* score than the combination of ET-KNN with hierarchical, *K*-means, and DBSCAN. The combination of KNN with fuzzy C-means also achieved 2%, 5%, and 6% higher *F* score than the combination of KNN with the hierarchical, *K*-means, and DBSCAN, while the SMO in combination with fuzzy C-means achieved 1%, 5%, and 7% higher *F* score than the combination of SMO with the hierarchical, *K*-means, and DBSCAN, respectively.

Table 12 shows the results on the Milan dataset using leave-one-day-out cross-validation. It demonstrates that the combination of fuzzy C-means with ANN achieved 3%, 6%, and 8% higher *F* score than the combination of hierarchical, *K*-means, and DBSCAN with ANN. ET-KNN with fuzzy C-means achieved 1%, 4%, and 8% higher *F* score than the combination of ET-KNN with hierarchical, *K*-means, and DBSCAN. The combination of KNN with fuzzy C-means also achieved 1%, 6%, and 8% higher *F* score than the combination of KNN with the hierarchical, *K*-means, and DBSCAN, while the SMO in combination with fuzzy C-means and hierarchical achieved 5% and 5% higher *F* score than the combination of SMO with the *K*-means and DBSCAN, respectively.

### 7.1. Confusion Matrix with Activities Balancing

Tables 9–12 show that the overall performance of ANN is much better than ET-KNN, KNN, and SMO when over-sampling method SMOTE is applied with fuzzy C-means, hierarchical, *K*-means, and DBSCAN. However, only confusion matrices of ANN in the combination of fuzzy C-means on both datasets, Aruba and Milan, are extracted again to compare the results. Through these confusion matrices, it analyzed that the performance of overlapping activities is much better than the previous results with imbalance activities and also from state-of-the-art study [23, 39, 40, 49]. Below, confusion matrices 13 and 14 show with the bold cells how instances of overlapping activities are correctly recognized now that were mixed before when activities were imbalanced.

Table 13 shows the confusion matrix on the Aruba dataset using threefold cross-validation in the combination of fuzzy C-means with ANN while activities are balanced. It shows that the recognition rate of “House Keeping” is 18% higher than imbalance activities, and only 2% of its instances are misclassified as “Eating,” which was 10% before balancing. The recognition rate of “Wash Dish” is 40% higher than imbalance activities, and only 10% of its instances are misclassified as “Meal Preparation,” which was 43% before balancing. The recognition rate of “Leave Home” is 36% higher than imbalance activities, and only 9% of its instances are misclassified as “Enter Home,” which was 45% before balancing. The recognition rate “Work” is 5% higher than imbalance activities. Also, the recognition rate of “Resperate” is 10% higher than imbalance activities, and only 8% of its instances are misclassified as “Work,” which was 15% before balancing.

Table 14 shows the confusion matrix on the Milan dataset using threefold cross-validation in the combination of fuzzy C-means with ANN while activities are balanced. It shows that the recognition rate of “Bed to Toilet” is 7% higher than imbalance activities, and only 7% of its instances are misclassified as “Master Bathroom,” which was 15% before balancing. The recognition rate of “Master Bathroom” is 7% higher than imbalance activities, and only 7% of its instances are misclassified as “Bed to Toilet,” which was 13% before balancing. The recognition rate of “Master Room” and “Read” is 10% and 4% higher than imbalance activities. The recognition rate of “TV” is 10% higher than imbalance activities, and only 4% of its instances are misclassified as “Read,” which was 10% before balancing. The recognition rate of “Morning Medicine” is 7% higher than imbalance activities, and only 6% of its instances are misclassified as “Kitchen Activity,” which was 10% before balancing. The recognition rate “Chores” is 10% higher than imbalance activities, and only 3% of its instances are misclassified as “Master Room,” which was 15% before balancing. The recognition rate of “Evening Medicine” is 17% higher than imbalance activities, and only 10% of its instances are misclassified as “Morning Medicine,” which was 21% before balancing. The recognition rate “Mediate” is 26% higher than imbalance activities, and only 4% and 4% of its instances are misclassified as “Morning Medicine” and “Evening Medicine,” which was 10% and 8% before balancing.

## 8. Discussion

This section explains “why fuzzy C-means with ANN shows better performance than other techniques.” We are dealing with the two-layer model for recognition: first, grouping similar activities from non-similar activities (the coarse-grained level), and secondly, correctly recognizing all different activities on a fine-grained level in a group of similar activities. Thus, the more accurate the grouping (clustering) level, the more accurately recognizing similar activities that share the same features. It is explained that fuzzy C-means clustering allows the piece of information to exist in more than one cluster based on probabilities, while the other clustering methods such as hierarchical, *K*-means, and DBSCAN allow info to be restricted in one cluster only. So, fuzzy C-means gives the advantage in our problem of overlapping activities' dataset. Also, ANN handles sparsity and uncertainty in overlapping datasets Aruba and Milan better than the ET-KNN, KNN, and SMO. Through subsections , it is concluded that fuzzy C-means make clusters better than hierarchical, *K*-means, and DBSCAN. Also, our approach achieved a 10% higher *F* score with the combination of fuzzy C-means and ANN with balanced activities than imbalance activities. This combination is our approach named overlapping activity recognition using clustering-based classification (OAR-CbC).

## 9. Comparison Study

We compare results of our approach “OAR-CbC” with state-of-the-art study [23, 39, 40, 49].  Table 15 shows that “OAR-CbC” achieved almost 13%, 18%, and 14% higher precision than [23, 39, 40], respectively. Our approach achieved 13%, 10%, and 16% higher recall than [23, 39, 40], respectively. Also, our approach achieved 14%, 16%, 18%, and 24% higher *F* score than [23, 39, 40, 49], respectively. Although the accuracy of [39] is 5% higher than our approach, the accuracy measure cannot be considered, when the dataset is imbalanced and the study [39] used imbalanced dataset. The study [39] extracted results with under-sampling data, so, for fair comparisons, we also extracted results with under-sampling. The proposed approach achieved 2% higher recall and *F* score than [39]. In case of default sampling, we achieved 9% and 5% higher precision and 2% and 8% higher recall than [23, 40], respectively. Also, we achieved 7%, 9%, and 15% higher *F* score than [23, 40, 49], respectively. The cells are highlighted with the bold text of [39, 40] in confusion matrices of Tables 16 and 17 in comparison with our approach of Table 13.  Table 16 of [40] demonstrates that the recognition rate of “House Keeping,” “Leave Home,” “Resperate,” and “Wash Dishes” is 8%, 80%, 24%, and 80% lower than our approach as in Table 13, respectively.  Table 17 of [39] demonstrates that the recognition rate of “Enter Home,” “House Keeping,” “Leave Home,” and “Wash Dishes” is 21%, 26%, 29%, and 85% lower than our approach as in Table 13, respectively.

The bar graph in Figure 3 illustrates the activity-level comparison results of OAR-CbC with the state-of-the-art study APMTA [23] and MkRENN [49] through *F* score on the Aruba dataset. Our approach attains a high *F* score in all the six overlapping activities compared with APMTA [23] and for all eleven activities compared with MkRENN [49], while it shows comparatively slightly less *F* score in “Sleep,” “Meal Preparation,” and “Relax” activity compared with APMTA [23]. From the detailed analysis of the proposed approach's results compared with the existing methods, it can be concluded that OAR-CbC proves to be more effective and reliable in recognizing overlapping activity instances.

## 10. Conclusion

Improving the recognition accuracy of activities with overlapping features in the smart home is significant because reliability is a major concern when these modules are applied to real-world problems to recognize complex activities. We analyze the similarity of activities and make a generic model to recognize activities with fewer interclass variations. Our clustering-based classification approach “OAR-CbC” works more robust than state-of-the-art research [23, 39, 40]. We extract results with clustering techniques fuzzy C-means [35], hierarchical [42], *K*-means [36], and DBSCAN [37] in combination with the classification methods ANN [45], ET-KNN [47], KNN [48], and SMO [46] on two smart home datasets Aruba and Milan in which activities are highly overlapped. The results stated that ANN gives better performance with fuzzy C-means of almost 85%, but the accuracy of some overlapping activities is 50%. After applied data balancing through SMOTE, ANN gives a higher score of almost 94% with 80%–90% accuracy of overlapping activities. Also, we analyze that other machine learning techniques used in extracting the results do not achieve better scores in case of overlapping activities as hierarchical achieves 90% for “Meal Preparation” but 50% for “Wash Dishes” even after data balancing. We ensured the reliability of our approach using different performance metrics. By improving the accuracy of one overlapping activity, “Wash Dish,” other relevant overlapping activity “Meal Preparation” performance decreases slightly by almost 5%. So, in future work, it could be addressed. Also, this generic model can be applied to other types of complex health activities.

## Figures and Tables

**Figure 1:** Block diagram of proposed approach.

**Figure 2:** Sample of raw and activity annotated sensor data. Sensors IDs starting with *M* are motion sensors.

**Figure 3:** Bar graph illustrating comparison results of OAR-CbC with the state-of-the-art study through *F* score on Aruba dataset. The range of the *F* score is between [0-1], with one being the highest. Key: OAR-CbC: proposed approach, APMTA [23], MkRENN [49], tlt: bed to toilet, eat: eating, EH: enter home, HK: housekeeping, LH: leave home, MP: meal preparation, Rlx: relax, Res: resperate, Slp: sleeping, WD: wash dishes, and WK: work.

**Table 1:** Comparative summary of state-of-the-art methods for activity recognition. All features mean no explicit features are selected.

References		[15]	[21]	[31]	[22]	[27]	[7]	[41]	[38]	[40]	[39]	[23]
Feature selection	All feature	✓	—	✓	—	✓	✓	✓	✓	—	✓	✓

Approach	Selected	—	✓	—	✓	—	—	—	—	✓	—	—
	*K*-means	✓	✓	—	—	—	—	—	—	✓	—	—
	HMM	✓	—	—	—	—	✓	—	✓	—	—	—
	CRF	—	—	—	—	—	✓	—	✓	—	—	—
	DCNN	—	—	—	—	—	—	—	—	—	✓	—
	VSM	—	—	—	—	—	—	—	—	—	—	✓
	DBSCAN	—	—	—	—	✓	—	✓	—	—	—	—
	SVM	—	✓	—	—	—	—	—	—	—	—	—
	D.S.T.o.E	—	—	—	✓	—	—	—	—	✓	—	—
	LDA	—	—	—	—	—	—	—	✓	—	—	—
	AdaBoost	—	—	—	—	—	—	—	✓	—	—	—
	NBC	—	—	✓	—	—	✓	—	—	—	—	—
	Itemset	—	—	—	—	✓	—	—	—	—	—	—

Datasets	CASAS	✓	—	—	—	—	✓	—	—	✓	✓	✓
	Kasteren	—	✓	—	—	✓	—	—	—	✓	—	✓
	SAD	—	—	—	—	—	—	—	✓	—	—	—
	UCI	—	—	—	—	—	—	—	✓	—	—	—
	HHAR	—	—	—	—	—	—	—	✓	—	—	—
	Self	—	—	✓	✓	—	—	✓	—	—	—	—

**Table 2:** Dataset summary.

Dataset	Activity name	Instances
Milan [34]	Bed_to_Toilet	89
	Chores	23
	Desk_Activity	54
	Dining_Rm_Activity	22
	Eve_Meds	19
	Guest_Bathroom	330
	Kitchen_Activity	554
	Leave_Home	214
	Master_Bathroom	306
	Meditate	17
	Watch_Tv	114
	Sleep	96
	Read	314
	Morning_Meds	41
	Master_Bedroom	117

Aruba [7]	Meal_Preparation	1606
	Relax	2910
	Eating	257
	Work	171
	Sleeping	401
	Wash_Dishes	65
	Bed_to_Toilet	157
	Enter_Home	431
	Leave_Home	431
	Housekeeping	33
	Resperate	6

**Table 3:** Performance evaluation metrics on the Aruba dataset without activities balancing using threefold cross-validation.

Dataset	Cross-validation	Clustering method	Classification method	Precision (%)	Recall (%)	*F* score [0,1]	Accuracy (%)
Aruba	Threefolds	Fuzzy C-means [35]	ANN [45]	**84.50**	**84.70**	**0.84**	**84.70**
			ET-KNN [47]	80.60	80.80	0.80	80.80
			KNN [48]	79.30	78.50	0.79	78.50
			SMO [46]	75.37	74.02	0.74	74.02
		Hierarchical [42]	ANN	82.80	83.80	0.82	83.80
			ET-KNN	80.80	80.70	0.80	80.80
			KNN	78.20	78.20	0.78	78.20
			SMO	76.02	75.01	0.74	76.02
		*K*-mean [36]	ANN	81.30	82.80	0.82	82.80
			ET-KNN	79.50	79.80	0.79	79.80
			KNN	77.50	78.20	0.78	78.20
			SMO	74.20	75.01	0.74	75.02
		DBSCAN [37]	ANN	79.20	80.80	0.80	80.80
			ET-KNN	78.30	78.80	0.78	78.80
			KNN	76.20	75.10	0.76	76.20
			SMO	74.02	74.02	0.74	74.02

The precision, recall, and accuracy are in percentages (%), while the range of *F* score is between [0-1] with 1 being the highest. The highest values are in bold.

**Table 4:** Performance evaluation metrics on Milan dataset without activities balancing using threefold cross-validation.

Dataset	Cross-validation	Clustering method	Classification method	Precision (%)	Recall (%)	*F* score [0, 1]	Accuracy (%)
Milan	Threefolds	Fuzzy C-means [35]	ANN [45]	**82.23**	**83.04**	**0.83**	**83.04**
			ET-KNN [47]	79.61	80.25	0.80	80.25
			KNN [48]	78.41	78.51	0.79	78.25
			SMO [46]	74.37	74.54	0.75	75.37
		Hierarchical [42]	ANN	80.01	81.01	0.81	81.01
			ET-KNN	77.51	77.91	0.78	78.01
			KNN	75.41	75.41	0.76	75.41
			SMO	73.23	72.22	0.72	73.23
		*K*-mean [36]	ANN	77.51	80.01	0.79	80.01
			ET-KNN	76.41	76.71	0.77	76.51
			KNN	74.71	75.41	0.76	75.41
			SMO	72.41	72.22	0.73	72.23
		DBSCAN [37]	ANN	78.41	78.51	0.79	78.71
			ET-KNN	76.51	77.01	0.77	77.01
			KNN	74.61	73.41	0.74	74.61
			SMO	72.31	73.41	0.73	73.51

The precision, recall, and accuracy are in percentages (%), while the range of *F* score is between [0-1], with 1 being the highest. The highest values are in bold.

**Table 5:** Confusion matrix on the Aruba dataset without activities balancing using threefold in combination of fuzzy C-means and ANN.

Acts	Slp	Tlt	MP	Rlx	HK	Eat	WD	LH	EH	WK	Res
Slp	97.9			2.1							
Tlt	2.7	97.2									
MP			95.2				3.1		1.7		
Rlx	1.8			97.6					0.6		
HK				5.1	**80.0**	**9.7**			5.2		
Eat			5.8	2.0		92.2					
WD			**43.9**	7.1			**50.0**				
LH								**55.0**	**45.0**		
EH								9.2	90.8		
WK				8.4						91.6	
Res						1.0				**18.0**	**81.0**

The columns represent the predicted activities, while the rows represent the actual activities. The performance of overlapping activities is highlighted in bold. *Key*. acts: activities, tlt: bed to toilet, eat: eating, EH: enter home, HK: housekeeping, LH: leave home, MP: meal preparation, Rlx: relax, Res: resperate, Slp: sleeping, WD: wash dishes, and WK: work.

**Table 6:** Confusion matrix on the Aruba dataset without activities balancing using threefold in combination of hierarchical and ANN.

Acts	Slp	Tlt	MP	Rlx	HK	Eat	WD	LH	EH	WK	Res
Slp	89.7	2.3		8.0							
Tlt	6.8	93.2									
MP			94.0			2.2	3.8				
Rlx	4.4			94.6		1.0					
HK			3.2	6.8	89.6	0.4					
Eat			4.4	16.4		86.4			2.8		
WD			**45.5**			**10.0**	**45.5**				
LH								**75.1**	**24.9**		
EH			3.0					**11.7**	**85.3**		
WK			1.8	9.8						85.2	3.2
Res						5.0				**15.0**	**80.0**

The columns represent the predicted activities, while the rows represent the actual activities. The performance of overlapping activities is highlighted in bold.

**Table 7:** Confusion matrix on the Milan dataset without activities balancing using threefold in the combination of fuzzy C-means and ANN.

Acts	Slp	Tlt	Dsk	Dnr	Gbr	Kch	Mbr	Lh	Mr	Red	Tv	Mmd	Chr	Emd	Med
Slp	86.4						1.3		7.4	2.6	2.3				
Tlt		**79.5**			5.4		**15.1**								
Dsk			83.3	4.5			3.2						9.0		
Dnr				83.8		10.3				1.2	4.7				
Gbr		9.5			85.5		5.0								
Kch						87.2	1.3					11.5			
Mbr	1.0	**13.7**			2.0		**83.3**		3.0						
Lh								98.0	2.0						
Mr	5.0						2.4		**83.0**	2.6	5.4		1.6		
Red									3.4	91.6	5.0				
Tv						2.3			4.7	**10.7**	**82.3**				
Mmd						**10.0**	4.8					**78.2**		7.0	
Chr						5.0			**15.0**		4.0		**76.0**		
Emd						8.3						**21.3**		**70.4**	
Med					2.5	4.5	5.2	4.8				8.1		**10.5**	**64.4**

The columns represent the predicted activities, while the rows represent the actual activities. The score of overlapping activities is highlighted in bold. *Key*. acts: activities, Slp: sleeping, Tlt: bed to toilet, Dsk: desk activity, Dnr: dining room activity, Gbr: guest bathroom, Kch: kitchen activity, Mbr: master bathroom, Lh: leave home, Mr: master bedroom, Red: read, Tv: watch Tv, Mmd: morning medicine, Chr: chores, Emd: evening medicine, and Med: mediate.

**Table 8:** Confusion matrix on the Milan dataset without activities balancing using threefold in the combination of hierarchical and ANN.

Acts	Slp	Tlt	Dsk	Dnr	Gbr	Kch	Mbr	Lh	Mr	Red	Tv	Mmd	Chr	Emd	Med
Slp	82.4							2.3	9.4	2.6	2.3				
Tlt		**75.5**			7.0		**17.5**								
Dsk			83.3	4.5					3.2				9.0		
Dnr				**80.8**		**13.3**				1.2	4.7				
Gbr		9.5			85.5		5.0								
Kch				1.0		86.2	1.3					11.5			
Mbr	2.0	**13.7**			3.2		**81.1**		3.0						
Lh						1.0		95.0	4.0						
Mr	6.0						2.4		80.0	3.6	6.4		1.6		
Red									3.7	91.3	5.0				
Tv						4.1			2.9	10.8	82.2				
Mmd						**10.0**	3.1					**74.9**		**12.0**	
Chr						5.0			**15.0**		4.0		**76.0**		
Emd						**10.3**						**22.5**		**67.2**	
Med					2.5	4.4	5.3	5.8	1.0			7.1		**11.5**	**60.4**

The columns represent the predicted activities, while the rows represent the actual activities. The performance of overlapping activities is highlighted in bold.

**Table 9:** Performance evaluation metrics on the Aruba dataset with activities balancing using threefold cross-validation.

Dataset	Cross-validation	Clustering method	Classification method	Precision (%)	Recall (%)	*F* score [0, 1]	Accuracy (%)
Aruba	Threefolds	Fuzzy C-means [35]	ANN [45]	**93.60**	**92.40**	**0.93**	**93.30**
			ET-KNN [47]	87.30	87.80	0.87	87.40
			KNN [48]	85.20	85.40	0.85	85.10
			SMO [46]	80.80	80.70	0.8	80.30
		Hierarchical [42]	ANN	88.20	88.80	0.88	88.50
			ET-KNN	85.20	85.30	0.85	85.30
			KNN	83.30	83.80	0.83	83.80
			SMO	79.50	79.50	0.79	79.20
		*K*-mean [36]	ANN	86.20	86.30	0.86	86.70
			ET-KNN	83.20	83.80	0.83	83.80
			KNN	80.40	80.30	0.80	80.20
			SMO	77.30	76.02	0.75	76.02
		DBSCAN [37]	ANN	83.30	83.80	0.83	83.80
			ET-KNN	80.20	80.40	0.80	80.20
			KNN	77.30	77.20	0.77	77.20
			SMO	76.02	76.02	0.76	76.10

The precision, recall, and accuracy are in percentages (%), while the range of *F* score is between [0-1] with 1 being the highest. The highest values are in bold.

**Table 10:** Performance evaluation metrics on the Aruba dataset with activities balancing using leave-one-day-out cross-validation.

Dataset	Cross-validation	Clustering method	Classification method	Precision (%)	Recall (%)	*F* score [0, 1]	Accuracy (%)
Aruba	Leave one day out	Fuzzy C-means [35]	ANN [45]	**94.30**	**94.10**	**0.94**	**94.40**
			ET-KNN [47]	88.20	88.50	0.88	88.10
			KNN [48]	86.10	86.20	0.86	86.10
			SMO [46]	81.40	81.20	0.81	81.40
		Hierarchical [42]	ANN	89.40	90.20	0.89	89.60
			ET-KNN	87.30	87.80	0.87	87.40
			KNN	85.50	85.10	0.85	85.10
			SMO	81.30	81.30	0.81	81.40
		*K*-mean [36]	ANN	87.60	87.10	0.87	87.20
			ET-KNN	84.80	85.40	0.85	85.10
			KNN	82.10	81.30	0.81	81.10
			SMO	77.30	77.20	0.77	77.20
		DBSCAN [37]	ANN	85.70	85.10	0.85	85.10
			ET-KNN	81.20	81.30	0.81	81.30
			KNN	79.10	79.10	0.79	79.50
			SMO	78.02	78.20	0.78	78.30

The precision, recall, and accuracy are in percentages (%), while the range of *F* score is between [0-1] with 1 being the highest. The highest values are in bold.

**Table 11:** Performance evaluation metrics on the Milan dataset with activities balancing using threefold cross-validation.

Dataset	Cross-validation	Clustering method	Classification method	Precision (%)	Recall (%)	*F* score [0, 1]	Accuracy (%)
Milan	Threefolds	Fuzzy C-means [35]	ANN [45]	**92.20**	**92.50**	**0.92**	**92.20**
			ET-KNN [47]	86.20	86.50	0.86	86.70
			KNN [48]	84.30	85.40	0.85	85.10
			SMO [46]	80.50	80.30	0.80	80.30
		Hierarchical [42]	ANN	89.30	89.40	0.89	89.40
			ET-KNN	85.20	85.30	0.85	85.30
			KNN	83.30	83.80	0.83	83.80
			SMO	79.40	79.10	0.79	79.50
		*K*-mean [36]	ANN	85.50	85.10	0.85	85.10
			ET-KNN	83.20	82.80	0.83	83.50
			KNN	79.70	80.30	0.80	80.50
			SMO	77.30	76.02	0.75	76.02
		DBSCAN [37]	ANN	83.30	83.80	0.83	83.80
			ET-KNN	80.20	80.40	0.80	80.20
			KNN	79.50	79.20	0.79	79.20
			SMO	78.02	78.20	0.78	78.30

The precision, recall, and accuracy are in percentages (%), while the range of *F* score is between [0-1] with 1 being the highest. The highest values are in bold.

**Table 12:** Performance evaluation metrics on the Milan dataset with activities balancing using leave-one-day-out cross-validation.

Dataset	Cross-validation	Clustering method	Classification method	Precision (%)	Recall (%)	*F* score [0, 1]	Accuracy (%)
Milan	Leave one day out	Fuzzy C-means [35]	ANN [45]	**93.40**	**93.20**	**0.93**	**93.30**
			ET-KNN [47]	89.30	89.40	0.89	89.40
			KNN [48]	87.10	87.20	0.87	87.10
			SMO [46]	83.30	83.80	0.83	83.80
		Hierarchical [42]	ANN	90.50	90.40	0.90	90.60
			ET-KNN	88.10	88.20	0.88	88.40
			KNN	86.20	86.50	0.86	86.70
			SMO	83.10	83.70	0.83	83.80
		*K*-mean [36]	ANN	87.60	87.10	0.87	87.20
			ET-KNN	84.30	85.20	0.85	85.50
			KNN	81.10	81.30	0.81	81.10
			SMO	78.02	78.20	0.78	78.30
		DBSCAN [37]	ANN	85.70	85.10	0.85	85.10
			ET-KNN	81.20	81.30	0.81	81.30
			KNN	79.10	79.10	0.79	79.50
			SMO	78.20	78.50	0.78	78.20

The precision, recall, and accuracy are in percentages (%), while the range of *F* score is between [0-1] with 1 being the highest. The highest values are in bold.

**Table 13:** Confusion matrix on the Aruba dataset with activities balancing using threefold in combination of fuzzy C-means and ANN.

Acts	Slp	Tlt	MP	Rlx	HK	Eat	WD	LH	EH	WK	Res
Slp	97.9	2.1									
Tlt		98.0		2.0							
MP			**85.2**	2.4		2.1	**10.2**				
Rlx	0.9		6.3	87.8		3.8			1.2		
HK					**98.3**	**1.7**					
Eat			4.0	2.0		93.0	1.0				
WD			**10.6**				**89.4**				
LH								**91.5**	**8.5**		
EH								**9.9**	**90.1**		
WK			1.1			2.1				96.4	
Res					1.0					**8.4**	**90.6**

The columns represent the predicted activities, while the rows represent the actual activities. The performance of overlapping activities is highlighted in bold. *Key*. acts: activities, Tlt: bed to toilet, Eat: eating, EH: enter home, HK: housekeeping, LH: leave home, MP: meal preparation, Rlx: relax, Res: resperate, Slp: sleeping, WD: wash dishes, and WK: work.

**Table 14:** Confusion matrix on the Milan dataset with activities balancing using threefold in the combination of fuzzy C-means and ANN.

Acts	Slp	Tlt	Dsk	Dnr	Gbr	Kch	Mbr	Lh	Mr	Red	Tv	Mmd	Chr	Emd	Med
Slp	96.2								3.8						
Tlt		**86.5**			4.0		7.5								
Dsk			94.0	2.8							1.2		2.0		
Dnr				**95.0**		**3.0**					2.0				
Gbr		4.2			93.0		2.6								
Kch				1.9		94.5			1.1			2.5	1.0		
Mbr		**7.0**					**90.0**		2.9						
Lh								100.0							
Mr							5.8		93.2				1.0		
Red						1.0				95.9	3.1				
Tv									3.7	4.0	92.3				
Mmd						**6.0**						**85.8**		**8.2**	
Chr						**9.6**			3.8				86.6		
Emd						**2.0**						**10.2**		**87.8**	
Med						2.1						**4.0**		**3.9**	**90.0**

The columns represent the predicted activities, while the rows represent the actual activities. The performance of overlapping activities is highlighted in bold. *Key*. acts: activities, Slp: sleeping, Tlt: bed to toilet, Dsk: desk activity, Dnr: dining room activity, Gbr: guest bathroom, Kch: kitchen activity, Mbr: master bathroom, LH: leave home, Mr: master bedroom, Red: read, Tv: watch Tv, Mmd: morning medicine, Chr: chores, Emd: evening medicine, and Med: mediate.

**Table 15:** Comparison results of our approach OAR-CbC with the state-of-the-art study.

Dataset	Cross-validation	Data sampling	Approach	Precision (%)	Recall (%)	*F*1 score [0, 1]	Accuracy (%)
Aruba	Threefold	Over-sampling	**OAR-CbC**	**93.60**	**92.40**	**0.93**	**93.30**
		Default sampling	**OAR-CbC**	**84.50**	**84.70**	**0.84**	**84.70**
	Tenfold	Under-sampling	**OAR-CbC**	**81.30**	**81.20**	**0.81**	**81.90**
			[39]	81.90	79.0	0.79	98.54
	Threefold	Default sampling	[23]	75.10	82.90	0.77	—
			[40]	79.65	76.46	0.75	91.40
			[49]	—	—	0.69	87.55

The precision, recall, and accuracy are in percentages (%), while the range of *F* score is between [0-1], with 1 being the highest. The highest values are in bold.

**Table 16:** Confusion matrix of paper [40] on the Aruba dataset using threefold cross-validation.

Acts	Tlt	Eat	EH	HK	LH	MP	Rlx	Res	Slp	WD	WK
Tlt	99.4						0.6				
Eat		94.2		0.4		2.3	3.1				
EH			95.8		3.5	0.7					
HK				90.9		3	6.1				
LH			**86.8**		**11.6**	1.2		0.2			
MP						96.8		0.6			2.3
Rlx		0.2		0.2		1.3	97.6		0.3		0.1
Res		0.4						**66.7**			**33.3**
Slp		0.3		0.2			1.5		**98.3**		
WD						**90.8**				**9.2**	
WK			0.6			0.6	1.8	0.6			96.5

The columns represent the predicted activities, while the rows represent the actual activities. The performance of overlapping activities is highlighted in bold.

**Table 17:** Confusion matrix of paper [39] on the Aruba dataset using tenfold cross-validation.

Acts	Tlt	Eat	EH	HK	LH	MP	Rlx	Slp	WD	WK
Tlt	100.0									
Eat		89.0		0.4		8.3	1.0			
EH	0.2		**69.1**	0.2	**30.5**					
HK			0.2	**72.5**		9.3	**16.2**	1.8		
LH			**36.9**	0.2	**62.7**	0.2				
MP		0.1		0.8		**98.1**	0.9		**0.2**	
Rlx				0.5		1.4	97.6	0.2		0.3
Slp			0.1	0.1	0.1		1.4	98.3		
WD						**96.0**			**4.0**	
WK				0.3		0.3	1.7			97.7

The columns represent the predicted activities, while the rows represent the actual activities. The performance of overlapping activities is highlighted in bold.

## Data Availability

Previously reported (sensor data for assessing human activities) data are used to support this study and are available at DOI: 10.1109/MIS.2010.112 and 10.3414/ME0592 or D. Cook's Learning setting-generalized activity models for smart spaces, IEEE Intelligent Systems, 2011, and D. Cook and M. Schmitter-Edgecombe's Assessing the quality of activities in a smart environment, Methods of Information in Medicine, 2009. These prior studies (and datasets) are cited at relevant places within the text as references [11, 16].
